# Neuromodulated Synaptic Plasticity on the SpiNNaker Neuromorphic System

**DOI:** 10.3389/fnins.2018.00105

**Published:** 2018-02-27

**Authors:** Mantas Mikaitis, Garibaldi Pineda García, James C. Knight, Steve B. Furber

**Affiliations:** ^1^Advanced Processor Technologies, Faculty of Science and Engineering, School of Computer Science, University of Manchester, Manchester, United Kingdom; ^2^Centre for Computational Neuroscience and Robotics, School of Engineering and Informatics, University of Sussex, Brighton, United Kingdom

**Keywords:** neuromodulation, STDP, SpiNNaker, three-factor learning rules, reinforcement learning, behavioral learning

## Abstract

SpiNNaker is a digital neuromorphic architecture, designed specifically for the low power simulation of large-scale spiking neural networks at speeds close to biological real-time. Unlike other neuromorphic systems, SpiNNaker allows users to develop their own neuron and synapse models as well as specify arbitrary connectivity. As a result SpiNNaker has proved to be a powerful tool for studying different neuron models as well as synaptic plasticity—believed to be one of the main mechanisms behind learning and memory in the brain. A number of Spike-Timing-Dependent-Plasticity(STDP) rules have already been implemented on SpiNNaker and have been shown to be capable of solving various learning tasks in real-time. However, while STDP is an important biological theory of learning, it is a form of Hebbian or unsupervised learning and therefore does not explain behaviors that depend on feedback from the environment. Instead, learning rules based on neuromodulated STDP (three-factor learning rules) have been shown to be capable of solving reinforcement learning tasks in a biologically plausible manner. In this paper we demonstrate for the first time how a model of three-factor STDP, with the third-factor representing spikes from dopaminergic neurons, can be implemented on the SpiNNaker neuromorphic system. Using this learning rule we first show how reward and punishment signals can be delivered to a single synapse before going on to demonstrate it in a larger network which solves the credit assignment problem in a Pavlovian conditioning experiment. Because of its extra complexity, we find that our three-factor learning rule requires approximately 2× as much processing time as the existing SpiNNaker STDP learning rules. However, we show that it is still possible to run our Pavlovian conditioning model with up to 1 × 10^4^ neurons in real-time, opening up new research opportunities for modeling behavioral learning on SpiNNaker.

## 1. Introduction

One of the earliest and most famous hypotheses on when synaptic plasticity occurs came from Donald Hebb, who postulated (Hebb, 1949):

“When an axon of cell A is near enough to excite a cell B and repeatedly or persistently takes part in firing it, some growth process or metabolic change takes place in one or both cells such that A's efficiency, as one of the cells firing B, is increased.”

In the context of the changing strengths of existing synaptic connections, rather than the formation of new synapses, Hebb's postulate suggests that connections between neurons whose activity is causally related will be strengthened. Neurons which persistently fire at the same time are likely to do so because they respond to similar or related stimuli.

Using improved experimental techniques that became available in the 1990s, Markram et al. (1997) showed that the magnitude of the changes in synaptic strength caused by Hebbian learning were related to the timing of pre- and post-synaptic spikes. The relationship between the magnitude of these changes and the relative timing of the pre- and post-synaptic spikes became known as Spike-Timing Dependent Plasticity (STDP) and the data recorded by Bi and Poo (1998) suggests that it reinforces causality between the firing of the pre- and post-synaptic neurons. When a pre-synaptic spike arrives before a post-synaptic spike is emitted the synapse is potentiated (strengthened). However, if a pre-synaptic spikes arrive after a post-synaptic spike has been emitted, the synapse is depressed (weakened). In the ensuing years STDP has been widely used to solve many tasks using biologically plausible spiking neural networks (Gerstner et al., 1996; Song et al., 2000; Davison and Frégnac, 2006).

Many extensions have been proposed to STDP such as the inclusion of additional spikes (Pfister and Gerstner, 2006) and the post-synaptic voltage (Brader et al., 2007; Clopath et al., 2010). However, while these extensions may improve the ability of STDP to capture the statistical relationship between pre- and post-synaptic activity, Hebbian learning still provides no means of controlling *what* to learn. For example, if we consider a two layer feed-forward network in which an output neuron is stimulated at the same time by two different input neurons, Hebbian learning will strengthen the synapses between both input neurons and the output. However, Hebbian learning rules provide no synapse-level means of associating reward or punishment; surprise or novelty; or any other input that could allow the system to learn how to behave in order to maximize reward. While circuit-level approaches such as attractor networks, built using only Hebbian learning rules (Amit, 1992; Giudice et al., 2003; Klampfl and Maass, 2013), can react differently to known and novel inputs, Hebbian learning rules cannot do this at a synaptic level. Dopamine (DA) has been identified as a potential reward signal in the brain (Schultz, 2000) and has been shown to control synaptic plasticity in a large number of ways (Shen et al., 2008). Also see Pawlak (2010) for a detailed review. On this basis Izhikevich (2007), Florian (2007), and Frémaux and Gerstner (2016) all developed learning rules based on *neuromodulation* which extend Hebbian learning to include reinforcement from neuromodulators such as dopamine.

SpiNNaker is a digital neuromorphic architecture designed for simulating spiking neural networks (Furber et al., 2014). SpiNNaker systems consist of varying numbers of custom SpiNNaker chips—each of which contains 18 simple, integer-only ARM cores which are connected through a network-on-chip and can communicate with their six neighboring chips using a multicast router. Each ARM core is typically programmed to simulate a number of neurons and communicates with the neurons simulated on other cores using spike events. Being able to define the neuron and synapse models in software makes SpiNNaker very flexible and has enabled a wide range of neuron models and integration methods (Hopkins and Furber, 2015) as well as synaptic plasticity algorithms (Jin et al., 2010; Galluppi et al., 2015; Lagorce et al., 2015; Knight et al., 2016) to been developed. Most recently Knight et al. (2016) developed a general framework, based on the algorithms developed by Morrison et al. (2007), for efficiently implementing STDP learning rules on SpiNNaker. Using this framework, Knight et al. successfully simulated large-scale models with tens of millions of plastic synapses on SpiNNaker.

Some progress has been made on simulating neuromodulated STDP on other neuromorphic hardware (Friedmann et al., 2013, 2017), but no large-scale networks using these learning rules have been demonstrated. In their technical report, Nichols et al. (2017) present the implementation of a three-factor learning rule for learning spatio-temporal patterns on SpiNNaker. However, in their learning rule, the third factor represents an attention signal—used to demarcate individual spatio-temporal patterns—rather than a biologically-inspired reinforcement signal. Additionally they only demonstrated this learning rule on small networks with up to 4 neurons and 1,000 input synapses.

While the methods we present in this paper could be used to simulate various three-factor learning rules on SpiNNaker, we demonstrate it in the context of the rule proposed by Izhikevich (2007), which we introduce in section 2.2. In section 2.1 we briefly outline the algorithm used to simulate STDP on SpiNNaker before, in section 2.3, we present an extended version of this algorithm which incorporates reward signals. In order to illustrate the functioning of this new algorithm, in section 3.1, we present the results of some simple network simulations which use reward and punishment signals to modulate learning. In section 3.2 we reproduce the classical conditioning experiment described by Izhikevich (2007) and use this to demonstrate both how neuromodulated STDP can be used to solve the credit assignment problem and how SpiNNaker can be used to simulate larger models incorporating neuromodulated STDP. Finally, in section 3.3, we measure the performance of our three-factor learning implementation—comparing the overhead with existing STDP models running on SpiNNaker and the run-time of the classical conditioning experiment with simulations running on GPU hardware with comparable energy requirements.

## 2. Materials and methods

### 2.1. Simulating STDP on SpiNNaker

STDP is simulated on SpiNNaker using a *trace-based* approach (Song et al., 2000; Morrison et al., 2008) where each synapse records pre- and post-synaptic neural activity into local trace variables (*s*_*i*_ and *s*_*j*_, respectively) with the following dynamics:

(1) $$\begin{array}{l} \frac{ds}{dt}=-\frac{s}{\tau }+\underset{t^{f}}{\sum }\delta \left(t-t^{f}\right), \end{array}$$

where spikes at times *t*^*f*^ – described by Dirac delta functions δ(*t*−*t*^*f*^)—increase the value of the trace which decays exponentially with a time constant τ. The time constants of these traces are typically set to match the shape of the desired STDP function.

Biological neurons have on the order of 10^3^–10^4^ afferent synapses, so updating all of these every time step would be extremely computationally intensive. Instead, as individual synapses only receive spikes at relatively low rates, they can be updated only when they transfer a spike as long as their new state can be calculated from their previous state.

Using this event-driven approach on SpiNNaker is also advantageous as, due to their sheer number, synapses need to be stored in the off-chip SDRAM which has insufficient bandwidth for every synapse's parameters to be retrieved every simulation time step (Painkras et al., 2013). Instead, synapses are updated only when spike packets arrive at a core and the row of the connectivity matrix associated with the pre-synaptic neuron is fetched from the off-chip SDRAM using a DMA transfer. Each row of the connectivity matrix describes the synapses going from a pre-synaptic neuron (the source of the spike) to a number of post-synaptic neurons.

Figure 1 illustrates how pre- and post-synaptic trace variables are sampled to compute STDP weight updates. This process is implemented using the *processRow()* function shown in Algorithm 1 which is called when a pre-synaptic spike arrives and the corresponding synaptic matrix row has been transferred into local memory. This algorithm applies all of the STDP updates that have occurred since the last pre-synaptic spike was received (between each pair of dashed blue vertical lines in Figure 1) in a similar manner to that proposed by Morrison et al. (2007). Firstly the spike times (*t*_*j*_) and associated trace values (*s*_*j*_) for each post-synaptic neuron connected by the synaptic row are retrieved from the post-synaptic history structure (located in the core's local memory). Then the effect of each post-synaptic spike (dashed green vertical lines in Figure 1) is applied to the synaptic weight using the *applyPostSpike* function. The effect of the pre-synaptic spike which triggered this update is then applied to the synaptic weight using the *applyPreSpike* function. Finally, the fully-updated weight is applied to the post-synaptic neural input (via a delay ring-buffer structure) using the *addWeightToRingBuffer* function. Once all of the synapses have been updated, the last pre-synaptic spike time (*t*_*old*_) and associated trace value (*s*_*i*_) stored in the synaptic row are updated.

**Figure 1:** Calculation of weight updates using pair-based STDP traces. Pre- and post-synaptic traces reflect spiking activity of pre- and post-synaptic neurons. Potentiation is calculated at each post-synaptic spike time by sampling the pre-synaptic trace (green circle) to obtain a measure of recent pre-synaptic activity. Depression is calculated at each pre-synaptic spike time by sampling the post-synaptic trace (blue circle) to obtain a measure of recent post-synaptic activity. Weight dependence is additive. After Morrison et al. (2008).

**Algorithm 1:** Algorithmic implementation of STDP (After Knight et al., 2016).

**function** processRow(*t*)
**for all** *j* **in** *postSynapticNeurons* **do**
*history* ← *getHistoryEntries*(*j, t*_*old*_, *t*)

**for all** (*t*_*j*_, *s*_*j*_) **in** *history* **do**
*w*_*ij*_ ← *applyPostSpike*(*w*_*ij*_, *t*_*j*_, *t*_*old*_, *s*_*i*_)

(*t*_*j*_, *y*_*j*_)←*getLastHistoryEntry*(*t*)
*w*_*ij*_ ← *applyPreSpike*(*w*_*ij*_, *t, t*_*j*_, *s*_*j*_)
*addWeightToRingBuffer*(*w*_*ij*_, *j*)

*s*_*i*_ ← *addPreSpike*(*s*_*i*_, *t, t*_*old*_)
*t*_*old*_ ← *t*

### 2.2. Neuromodulated-STDP model

Izhikevich explains that dopamine-modulated STDP has a built-in instrumental conditioning property, i.e., the associations between cues, actions and rewards are learned automatically by reinforcing the firing patterns (networks of synapses) responsible, even when the firings of those patterns are followed by a delayed reward or masked by other network activity. To achieve this each synapse has an *eligibility trace C*:

(2) $$\begin{array}{l} \frac{dC}{dt}=-\frac{C}{\tau_{c}}+STDP\left(\Delta t\right)\delta \left(t-t_{pre/post}\right), \end{array}$$

where τ_*c*_ is the decay time constant of the eligibility trace and *STDP*(Δ*t*) represents the magnitude of the change to make to the eligibility trace in response to a pair of pre- and post-synaptic spikes with temporal difference Δ*t* = *t*_*post*_ − *t*_*pre*_. Finally, δ(*t* − *t*_*pre*/*post*_) is a Dirac delta function used to apply the effect of STDP to the trace at the times of pre- or post-synaptic spikes.

The concentration of Dopamine is described by a variable *D*:

(3) $$\begin{array}{l} \frac{dD}{dt}=-\frac{D}{\tau_{d}}+D_{c}\underset{t_{d}^{f}}{\sum }\delta \left(t-t_{d}^{f}\right), \end{array}$$

where τ_*d*_ is the time constant of dopamine re-absorption, *D*_*c*_ is the increase in dopamine concentration caused by each incoming dopaminergic spike and $t_{d}^{f}$ are the times of these spikes.

Equations (2, 3) are then combined to calculate the change in synaptic strength *W*:

(4) $$\begin{array}{l} \frac{dW}{dt}=CD. \end{array}$$

As discussed in section 1, when a post-synaptic spike arrives very shortly after a pre-synaptic spike, a standard STDP rule would immediately potentiate the synaptic strength. However, as Figure 2 illustrates, when using the three-factor STDP rule, this potentiation would instead be applied to the eligibility trace. Because changes to the synaptic strength are gated by dopamine concentration *D* (Equation 4), changes are only made to the synaptic strength if *D* ≠ 0. Furthermore, if the eligibility trace has decayed back to 0 before any dopaminergic spikes arrive, the synaptic strength will not be changed.

**Figure 2:** Using eligibility trace *C* to gate STDP with dopamine *D*. After Izhikevich (2007).

### 2.3. Simulating neuromodulated-STDP on SpiNNaker

Because Equation (4) describes a continuous weight change, it cannot be directly evaluated within the event-driven STDP algorithm described in section 2.1. However, in this section we will show how it can be transformed into a form suitable for event-driven evaluation. Firstly we consider the *C* and *D* traces (Equations 2, 3). Similarly to the pre- and post-synaptic STDP traces discussed in section 2.1, between the times at which spikes occur, both of these equations are simple first-order linear ODEs. Therefore, we can write down the following equations to update *C* and *D*:

(5) $$\begin{array}{l} C_{ij}=C_{ij}\left(t_{c}^{last}\right)e^{-\frac{t-t_{c}^{last}}{\tau_{c}}}, \end{array}$$

(6) $$\begin{array}{l} D_{j}=D_{j}\left(t_{d}^{last}\right)e^{-\frac{t-t_{d}^{last}}{\tau_{d}}}, \end{array}$$

where $t_{c}^{last}$ is the time of the last eligibility trace update (when either a pre- or post-synaptic spike caused an STDP update) and $t_{d}^{last}$ is the time of the last dopamine trace update (occurs when a dopamine spike is received). So that each (post-synaptic) neuron can be independently targeted by dopaminergic spikes, the dopamine trace values (*D*) are stored in the post-synaptic history structure along with the post-synaptic traces (*s*_*j*_) and event times (*t*_*j*_) in a similar manner to the “target spikes” in the learning rule presented by Nichols et al. (2017). However, because the eligibility traces (*C*) are individual to each synapse, they must be stored alongside the synaptic weights (*w*_*ij*_) in SDRAM and can thus only be updated within the *processRow* function when have been transferred into local memory. We can now substitute Equations (5, 6) into Equation (4) to obtain the weight change dynamics:

(7) $$\begin{array}{l} \frac{dw_{ij}}{dt}=C\left(t_{c}^{last}\right)D\left(t_{d}^{last}\right)e^{-\frac{t-t_{c}^{last}}{\tau_{c}}}e^{-\frac{t-t_{d}^{last}}{\tau_{d}}}. \end{array}$$

Now, by integrating the preceding equation, the total weight change since the last update at *t*_*last*_ can be found:

(8) $$\begin{array}{l} \Delta w_{ij}=C\left(t_{c}^{last}\right)D\left(t_{d}^{last}\right)\int_{t^{last}}^{t}e^{-\frac{t-t_{c}^{last}}{\tau_{c}}}e^{-\frac{t-t_{d}^{last}}{\tau_{d}}}dt, \end{array}$$

(9) $$\begin{array}{l} \Delta w_{ij}=\frac{C\left(t_{c}^{last}\right)D\left(t_{d}^{last}\right)}{-\left(\frac{1}{\tau_{c}}+\frac{1}{\tau_{d}}\right)}\left(e^{-\frac{t-t_{c}^{last}}{\tau_{c}}}e^{-\frac{t-t_{d}^{last}}{\tau_{d}}}-e^{-\frac{t^{last}-t_{c}^{last}}{\tau_{c}}}e^{-\frac{t^{last}-t_{d}^{last}}{\tau_{d}}}\right). \end{array}$$

The final update Algorithm 1 makes to each synaptic weight is to apply the effect of the pre-synaptic spike at time *t*. Therefore, if we extend Algorithm 1 to update the eligibility trace, *t*_*old*_ will always represent the last time *C* was updated i.e., $t^{last}=t_{c}^{last}=t_{old}$. Furthermore, before the inner loop over the post-synaptic events occurs, we can decay the last dopamine trace value to *t*_*old*_ using Equation (6). Therefore, $t^{last}=t_{d}^{last}=t_{c}^{last}=t_{old}$, meaning that Equation (9) can be simplified to:

(10) $$\begin{array}{l} \Delta w_{ij}=\frac{C\left(t_{old}\right)D\left(t_{old}\right)}{-\left(\frac{1}{\tau_{c}}+\frac{1}{\tau_{d}}\right)}\left(e^{-\frac{t-t_{old}}{\tau_{c}}}e^{-\frac{t-t_{old}}{\tau_{d}}}-1\right). \end{array}$$

Algorithm 2 shows the extended, three-factor STDP algorithm. The *applyPostSpike* and *applyPreSpike* functions used to directly update the synaptic weight in Algorithm 1 are now instead used to update the eligibility trace (*C*_*ij*_). When pre- or post-synaptic events are applied, Equation (5) is used to decay the eligibility trace (*C*_*ij*_) and Equation (10) is used to update the synaptic weight (*w*_*ij*_). Finally, as previously discussed, Equation (6) is used to obtain the decayed *D*_*j*_ trace values at *t*_*old*_ and *t*.

**Algorithm 2:** Algorithmic implementation of three-factor STDP.

**function** processRow(*t*)
**for all** *j* **in** *postSynapticNeurons* **do**
*history* ← *getHistoryEntries*(*j, t*_*old*_, *t*)
(*t*_*prev*_, *s*_*prev*_, *D*_*prev*_, *type*_*prev*_) ← *getPrecedingHistoryEntry*(*t*)
*t*_*c*_ ← *t*_*old*_
$D_{c}\leftarrow D_{prev}exp\left(\frac{-(t_{c}-t_{prev}}{\tau_{D}}\right)$
**for all** (*t*_*j*_, *s*_*j*_, *D*_*j*_, *type*_*j*_) **in** *history* **do**
$w_{ij}\leftarrow w_{ij}+\frac{C_{ij}D_{c}}{-\left(\frac{1}{\tau_{C}}+\frac{1}{\tau_{D}}\right)}\left(exp\left(-\frac{(t_{j}-t_{c}}{\tau_{C}}\right)exp\left(-\frac{(t_{j}-t_{c}}{\tau_{D}}\right)-1\right)$
$C_{ij}\leftarrow C_{ij}exp\left(-\frac{t_{j}-t_{c}}{\tau_{C}}\right)$
**if** *type*_*j*_ **is not** *dopamine* **then**
*C*_*ij*_ ← *applyPostSpike*(*C*_*ij*_, *t*_*j*_, *t*_*old*_, *s*_*i*_)
*D_c_* ← *D*_*j*_
*t*_*c*_ ← *t*_*j*_

(*t*_*j*_, *s*_*j*_, *D*_*j*_, *type*_*j*_)←*getLastHistoryEntry*(*t*)
$w_{ij}\leftarrow w_{ij}+\frac{C_{ij}D_{c}}{-\left(\frac{1}{\tau_{C}}+\frac{1}{\tau_{D}}\right)}\left(exp\left(-\frac{(t-t_{c}}{\tau_{C}}\right)exp\left(-\frac{(t-t_{c}}{\tau_{D}}\right)-1\right)$
$C_{ij}\leftarrow C_{ij}exp\left(-\frac{t-t_{c}}{\tau_{C}}\right)$
*C*_*ij*_ ← *applyPreSpike*(*C*_*ij*_, *t, t*_*j*_, *s*_*j*_)
*addWeightToRingBuffer*(*w*_*ij*_, *j*)

*s*_*i*_ ← *addPreSpike*(*s*_*i*_, *t, t*_*old*_)
*t*_*old*_ ← *t*


In order to allow users to describe dopaminergic synapses we modified sPyNNaker (Stokes et al., 2017), the SpiNNaker implementation of PyNN (Davison et al., 2009) to support dopaminergic connections. To implement the dopamine signal we introduced dopaminergic neurons that communicate through a special type of synapses (similar to the “target synapses” employed by Nichols et al., 2017) which do not cause updates to the membrane potential of the post synaptic neuron but simply bring information about dopaminergic spikes into it. This approach has the advantage of allowing any type of PyNN neuron to act as a source of dopaminergic spikes. When a core receives a dopaminergic spike it is not added to the delay ring-buffer but is instead added directly to the post synaptic history structure where they can be accessed by Algorithm 2.

## 3. Results

### 3.1. Reinforcing a synapse on SpiNNaker

In this section we first demonstrate how the magnitude of synaptic weight changes caused by the learning rule described in section 2.2 depends on the delay preceding a “reward” or “punishment” reinforcement signal. Figure 3 shows the result of an experiment where reinforcement signals with different delays are injected after a pre-post spike pair (separated by 1 ms). When a reinforcement signal is introduced after a small delay of 4 ms, it produces a large change in synaptic strength as the eligibility trace has not had time to decay. However, if the reinforcement signal is delayed by a larger time, the eligibility trace will have decayed significantly and the change in synaptic strength will be much smaller. Furthermore, once the eligibility trace has decayed to 0, even if a reinforcement signal is received, the synaptic strength will remain unchanged (as dictated by Equation 4).

**Figure 3:** The strength of a single synapse after delayed reward and punishment. Each data point represents a separate experiment with a single pre-synaptic neuron connected to two post-synaptic neurons. A single pre-synaptic spike at time 1 ms is fired which causes both post-synaptic neurons to fire at time 3 ms. A single dopaminergic spike with *D*_*c*_ = 0.1 for reward and *D*_*c*_ = −0.1 for punishment is fired at different times between 4 and 3,000 ms. All the parameters are set to the values shown in Tables 1, 2. It can be seen that the longer dopamine is delayed, the more the eligibility trace decays and thus the smaller the resultant weight change. When the eligibility trace decays to zero at around 2,400 ms, the synapses are no longer affected by dopamine release.

In Figure 4 we show the spiking activity of 10 neurons whose input synapses use the learning rule presented in section 2.2. We performed this experiment using a SpiNNaker simulation in which each of these 10 neurons receives input from an independent 50 Hz Poisson spike source. Additionally, a single dopamine spike source is connected to all 10 neurons. The synapses connecting the Poisson spike sources to the neurons were initialized with a weight of 1.5 nA. This causes the neurons to fire initially at a low rate in response to the Poisson input but, when reward signals (green arrows) are applied to these synapses, the firing rate of all 10 neurons increases. However, when punishment signals (red arrows) are applied to these synapses, the neurons' firing rate reduces to the point that some stop firing, depending on magnitudes of eligibility traces at the times of punishment signal. An example usage of such a setup would be for the online training of a neural motor-control circuit where reinforcement signals could be used to modify the strengths of the synapses that drove the current motor output so as to fine-tune its magnitude.

**Figure 4:** Ten neurons connected to 10 Poisson spike sources, each with a mean firing rate of 50 Hz. Dopamine is injected at times 2,000 ms, 3,000 ms, and 4,000 ms (Green markers). This causes potentiation of synaptic connections between stimuli and post-synaptic neurons which causes post-synaptic neurons to respond more strongly. We then apply punishment (negative dopamine value, red markers) at times 8,000 ms, 9,000 ms, 10,000 ms which causes a reduced response to the same random stimuli. The experiment was performed with parameters τ_*d*_ = 5.0 ms, τ_*c*_ = 100.0 ms; reward signals were represented using *D*_*c*_ = 0.01; and punishment signals using *D*_*c*_ = −0.002. Due to Poissonian stimulus and short timing constants for eligibility and dopamine traces, not all synapses get potentiated. On the other hand, punishment is more effective because spiking rate is higher and thus eligibility traces have non-zero values constantly.

### 3.2. Solving the credit assignment problem on SpiNNaker

Pavlov and Thompson (1902) first described classical conditioning: a phenomenon in which a biologically potent stimulus–the *Unconditional Stimulus (UC)*—is initially paired with a neutral stimulus—the *Conditional Stimulus CS*). After many trials, learning is observed when the previously neutral stimuli starts to elicit a response similar to that which was previously only elicited by the biologically potent stimulus. Pavlov and Thompson performed many experiments with dogs, observing their response (by monitoring salivation) to the appearance of a person who has been feeding them and the actual food appearing (UC). He demonstrated that the dogs started to salivate in the presence of the person who has been feeding them (or any other CS), rather than just when the food appears, because the CS had previously been associated with food.

While Pavlovian conditioning has been demonstrated in small networks of spiking neurons with Hebbian learning (Hofstoetter et al., 2005), in more realistic situations where there is a long delay between the stimuli and the reward and there is distracting network activity, it becomes impossible to determine which firing patterns from which neurons are responsible for the reward. This is known as the *credit assignment* or *distal reward* problem—brute-force solutions to which would require recording all spiking activity and, when a reward signal arrives, searching this data to find the synapses responsible for the reward. Fortunately, as Izhikevich (2007) described, the learning rule discussed in section 2.2 enables us to solve the credit assignment problem in networks of any size with minimal memory overhead and no requirement to search through synaptic data.

Izhikevich (2007) demonstrated a Pavlovian conditioning experiment in which a CS (*S*_1_) is repeatedly injected into the sea of random neural activity and then followed by a reward, which reinforces the neural pathways going from neurons representing *S*_1_. To simulate the experiment, 100 random sets of 50 neurons (each representing stimuli *S*_1_…*S*_100_) are chosen from the pool of 1,000 neurons. To deliver these stimulus to the network, we stimulated the 50 neurons representing the chosen stimulus by injecting a 1 ms pulse of super-threshold current. Next, a continuous input stream is formed consisting of stimuli *S*_*k*_(1 ≤ *k* ≤ 100) in a random order with random intervals between 100 and 300 ms. After every presentation of *S*_1_ a reward in the form of an increase of extra-cellular dopamine is delivered to all plastic synapse in the network after a random delay of up to 1 s. The delay is large enough to allow a few irrelevant input stimuli to be presented during the waiting period—these can be considered as distractors. At the beginning of the experiment the neurons representing each stimuli *S*_*k*_(1 ≤ *k* ≤ 100) respond equally. However, after many trials, the network starts to show reinforced response to the CS (*S*_1_). Because synapses coming out of neurons representing *S*_1_ are always tagged with the eligibility trace when the reward is delivered, whereas the synapses connected to neurons representing irrelevant stimuli will only be occasionally tagged, the average strength of synaptic connections from neurons representing stimuli *S*_1_ becomes stronger than the mean synaptic connection strength in the rest of the network. Therefore, the other neurons in the network learn to listen more closely to the stimuli *S*_1_, because the activation of this pathway causes a reward.

We reproduced Izhikevich's experiment on SpiNNaker using the three-factor learning rule presented in section 2.2. Our experimental set-up consists of a population with *N*_*T*_ Leaky Integrate-and-Fire (LIF) neurons, which are divided into 80% regular- and 20% fast-spiking (RS and FS, respectively); Table 1 shows the parametrization for each type. All neurons—modeled using the PyNN IF_curr_exp model (Davison et al., 2009)—connect to each other with 10% probability. Connections originating from RS neurons are excitatory and permit synaptic weight changes through dopamine-modulated STDP (Table 2) and FS neurons project through fixed inhibitory synapses.

**Table 1:** IfCurrExp Neuron model parameters for the PyNN simulation.

**Type/Param**	***C*_*m*_**	***I*_*offset*_**	**τ_*m*_**	**τ_*refrac*_**	**τ_*syn*_*E*_**	**τ_*syn*_*I*_**	***V*_*reset*_**	***V*_*rest*_**	***V*_*thresh*_**
	**[nF]**	**[nA]**	**[ms]**	**[ms]**	**[ms]**	**[ms]**	**[mV]**	**[mV]**	**[mV]**
Excitatory (RS)	0.3	0.005	10	4	1	1	−70	−65	−55.4
Inhibitory (FS)	0.3	0	10	2	1	1	−70	−65	−56.4

**Table 2:** STDP parameters.

**Parameter**	***A*_+_**	***A*_−_**	**τ_+_ [ms]**	**τ_−_[ms]**	**τ_*c*_ [ms]**	**τ_*d*_ [ms]**
Value	1	1	10	12	1,000	200

We designated $N_{g}=\frac{N_{T}}{10}$ (e.g., when $N_{T}=10^{3},\;N_{g}=100$) neural groups, with each group including $N_{pg}=\frac{N_{T}}{20}$ (e.g., when $N_{T}=10^{3},\;N_{pg}=50$) randomly selected neurons. Dopamine is delivered by a single neuron which projects to all of the neurons in the main population and, throughout the experiment, each neuron in the population is stimulated with a 10 Hz Poisson noise input. In Figure 5 we demonstrate the results of this experiment with *N*_*T*_ = 1, 000 (which corresponds to the third column in Table 3). Figure 5A shows that, over the course of 60 min of simulated time, the average strength (weight) of synapses coming from the neurons representing *S*_1_ gradually becomes greater than the average strength of all synapses in the network. In the early stages of the experiment the network responds similarly to all five randomly selected stimuli meaning that the network response to the neurons representing *S*_1_ being stimulated is indistinguishable from the response to other stimuli. However, after an hour of simulation, we can observe an increase in the activity of the neurons representing *S*_1_ when this stimuli is delivered (Figure 5C)—showing that these neurons been selectively associated. Finally, based on this increased response to *S*_1_, we can observe that the network learns which of the 100 stimuli brings rewards—even though the activity of the neurons representing *S*_1_ is masked by distracting spiking activity and the reward is delayed for up to 1 s. Therefore, as Izhikevich (2007) reported, injection of a global dopaminergic signal into the network allows it to identify a group of neurons responsible for the rewards even in the presence of Poisson noise and unrelated activity from other groups.

**Figure 5:** **(A)** Shows the average synaptic weight of synapses from the group of neurons representing *S*_1_ (green) and every synapse in the network (blue) for the first hour of the experiment. Randomly selected stimuli *S*_*k*_ are delivered to the network (black arrows), separated by random intervals of between 100 and 300 ms. These are visible in the synchronous spikes in **(B,C)**. Every time *S*_1_ is chosen, dopamine is delivered to the network (dashed line). Raster plot **(B)** depicts the first 1 s of network activity when *S*_1_ was delivered to the network; and **(C)** illustrates 1 s of activity after 1 h of simulation, showing how the neurons stimulated by *S*_1_ have learned to respond more strongly. Note that in **(A)**, the average of all the weights is increasing because, additionally to *S*_1_ always being rewarded, some stimuli *S*_*k*_ ≠ *S*_1_ also randomly get picked up soon before or after reward is delivered to the network.

**Table 3:** Effects of scaling conditioning network.

Neurons per core	90	90	90	90	90	90	60	60
Total neurons *N*_*T*_	200	500	1,000	2,000	4,000	6,000	8,000	10,000
Total synapses	4 K	25 K	100 K	400 K	1.6 M	3.6 M	6.4 M	10 M

In order to evaluate the scaling properties of our algorithm, we also simulated this network at the scales listed in Table 3 up to 10,000 neurons and 10 million synapses (keeping the connection probability and *N*_*g*_ constant). We found that the SpiNNaker system was able to simulate the experiment in real time at all of the listed network sizes. However, when the total number of neurons in the network reached 8,000, the increase in the number of incoming synapses per neuron required that we reduce the number of neurons simulated on each core to maintain real-time performance.

### 3.3. Performance

In this section we discuss performance statistics obtained by benchmarking the three-factor STDP learning rule running on SpiNNaker.

#### 3.3.1. Incoming spike processing performance

SpiNNaker machines have no form of global synchronization. Therefore, each core needs to update the state of each neuron it is responsible for simulating and process any incoming spikes it has received within a predetermined simulation time step (typically 1 ms). This means that the number of neurons simulated on each core, the complexity of the neuron or synapse model, the density of connectivity and the rate of incoming spikes all need to be balanced to guarantee real time operation.

In Figure 6 we compare the incoming spike processing performance of a single SpiNNaker core simulating a population of leaky-integrate-and-fire neurons with standard STDP and three-factor STDP synapses. The extra local memory required to store dopamine trace values in the post-synaptic history structure means that, when using the three-factor STDP algorithm described in section 2.3, each core is limited to simulating 126 neurons. As Knight and Furber (2016) discussed, the length of synaptic matrix rows has a significant effect on synapse processing performance. This is because, beyond the computational cost of processing each synapse, there is a large fixed cost in processing each row meaning that the best performance is obtained with long row lengths. Therefore, following the procedure outlined by Knight and Furber, we stimulated our population of neurons with an increasing number of 10 Hz Poisson spike trains in order to determine the maximum incoming spike rate that the core could process in real time. Additionally, because the number of events in the post-synaptic history structure affects the performance of Algorithms 1 and 2, we varied the post-synaptic firing rate by injecting a fixed current into the simulated neurons. Because, in the case of three-factor STDP, incoming dopaminergic spikes also get added to the post-synaptic history structure, we also measured the performance with a single dopaminergic neuron, firing at 8 Hz, connected to all the neurons in the benchmark population.

**Figure 6:** Comparison between incoming spike processing performance of standard STDP (with an additive weight dependence) and three-factor STDP for different post-synaptic spiking rates.

We find that the highest number of inputs into a single core can be achieved with rows approximately 60 synapses long (50 % connection density). Furthermore, as the post synaptic rate is increased, more synaptic history traces have to be processed on each pre-synaptic spike, so overall performance decreases. As predicted, we also find that performance with short synaptic rows (10–40 synapses per neuron) suffers from the fixed row-processing overheads mentioned earlier in this section. It is also worth noting that with very long synaptic rows (80–120 synapses per neuron) performance is also reduced. We predict that this is because, with very long rows that take a long time to process, even small variations in the number of spikes emitted by the Poisson sources each time-step can overrun the time available. The maximum number of inputs into a core simulating a network spiking at 10 Hz and neuromodulated with an 8 Hz dopaminergic signal was 0.38 million which is approximately two times slower than the simplest additive STDP rule.

#### 3.3.2. Moving toward cortical levels of connectivity

SpiNNaker was designed around the assumption that each ARM core would be responsible for simulating 1,000 neurons with 1,000 input synapses, each receiving spikes at a mean rate of 10 Hz (Jin et al., 2008). However, over recent years, it has been found that, on average, cortical neurons have 8,000 input synapses (Beaulieu and Colonnier, 1989; Pakkenberg et al., 2003; Braitenberg and Schüz, 2013) each receiving spikes at the lower average rate of around 3 Hz (Buzsaki and Mizuseki, 2014). While Knight and Furber (2016) showed that SpiNNaker was capable of simulating neurons in real-time with these higher levels of connectivity, even when using standard STDP this required reducing the number of neurons simulated on each core to only around 30. The alternative is to slow down the simulation to some fixed fraction of real-time. In Figure 7 we demonstrate how the number of neurons per core and the simulation speed can be traded off when simulating neurons with three-factor STDP and cortical levels of connectivity. Each neuron in the network is densely connected to 8,000 Poisson sources firing at 3 Hz as well as to a single dopaminergic neuron spiking at an average rate of 4.5 Hz. We found that, in order to simulate this network in real-time, the maximum number of neurons that could be simulated on each core was only 15. However, when we increased the number of neurons simulated on each core to the maximum of 126, we had to slow the simulation down by a factor of 11x.

**Figure 7:** Time to simulate 5 s of network activity with 8,000 inputs to each neuron. The mean firing rate of each input is 3 Hz, the post synaptic firing rate is 3 Hz, and the mean firing rate of the dopaminergic neuron is 4.5 Hz.

#### 3.3.3. Neuromodulated-STDP on SpiNNaker vs. GPUs

Neuromorphic architectures such as SpiNNaker have been specifically designed for the low-power simulation of spiking neuron networks. However, GPU architectures, although initially designed for accelerating the rendering of 3D graphics, have evolved into versatile accelerators which have been used in a wide range of HPC applications (Fan et al., 2004; Kindratenko et al., 2009)—notable deep-learning (Chellapilla et al., 2006; Cireşan et al., 2010). Additionally, with the demands of edge computing (Shi et al., 2016), GPUs are increasingly becoming available in form factors with comparable power requirements to neuromorphic hardware. One device of this type is the Jetson TX1, an embedded system with a peak power usage of only 18 W, yet still equipped with a 256 CUDA core “Maxwell” GPU as well as a 64 bit quad-core ARM Cortex-A57 and 4 GiB of LPDDR4 memory. Similarly to other GPU devices, the NVIDIA Jetson TX1 can be programmed using the Compute Unified Device Architecture (CUDA), meaning that a wealth of scientific software can be compiled for it including GeNN (Yavuz et al., 2016)—a code generation framework for spiking neural network simulations.

In this section we compare the performance of the Pavlovian conditioning experiment running on SpiNNaker that we presented in section 3.2 with the same model running on the Jetson TX1 using the GeNN simulator. Diamond et al. (2016) previously compared the performance of GeNN and SpiNNaker running a classification task but, although their model also used three-factor learning, Diamond et al. did not implement the learning rule on either SpiNNaker or GeNN. Instead Diamond et al. used standard STDP with a post-synaptic teaching signal on SpiNNaker and, when using GeNN, they performed learning on the host machine's CPU. However, based on Equation (9), we implemented a GeNN version of the dopamine modulated STDP rule described in section 2.2 so can provide a somewhat closer comparison. Furthermore, Diamond et al. (2016) compared SpiNNaker to an NVIDIA Titan Black—a high-end gaming card which uses up to 250 W of power—whereas the Jetson TX1's peak power usage of 18 W is much more comparable to the 26–36 W consumed by a 48 chip SpiNNaker system (Stromatias et al., 2013) making this an interesting comparison.

As discussed in section 3.2, we were able to run the Pavlovian conditioning experiment in real-time at all scales on SpiNNaker. However, GeNN simply runs the simulation as fast as possible and, as Figure 8 shows, when simulating this model simulation times increase approximately linearly with the number of synapses. Using the NVIDIA profiling tools to further analyse the performance suggests that the majority of time (88 % in the 10 × 10^3^ neuron model) is spent in the CUDA kernel responsible for applying weight updates resulting from post-synaptic spikes. Yavuz et al. (2016) also identified this as a bottleneck on mobile GPUs and suggested that this is due to the non-coalesced memory accesses that this kernel employs.

**Figure 8:** Time to simulate 1 h of the Pavlovian conditioning experiment described in section 3.2 at three different scales. SpiNNaker can simulate all configurations in real-time. The Jetson TX1 GPU and all CPUs are set to run at the maximum supported frequency.

## 4. Discussion

### 4.1. Reinforcement learning

Reinforcement learning is a biologically inspired learning paradigm where an agent learns by interacting with the world around it and modifies its behavior based on sparse feedback (for example a reward signal). Reinforcement learning has been shown to work effectively in convolutional neural networks (Mnih et al., 2015). However, it remains unclear how these techniques could be replicated in spiking neural networks and whether classical reinforcement learning (Sutton and Barto, 1998) is at all analogous to dopamine modulated synaptic plasticity in the brain (Reynolds et al., 2001; Pawlak and Kerr, 2008).

Bridging the gap between classical reinforcement learning and synaptic plasticity could be key to understanding, and using, low power neuromorphic systems, eventually simulating the human brain at scales not currently possible even on super computers. *Temporal Difference learning* is one of the most common reinforcement learning algorithms (Sutton and Barto, 1998) and some similarities between it and plasticity in the brain have been already observed (O'Doherty et al., 2004). Potjans et al. (2009) provided further evidence to support this link using a reinforcement learning framework implemented using a spiking neural network. In this framework reward is modeled as a real-valued signal which, rather than gating weight updates in the manner we describe in section 2.2, is simply added to the weight alongside any changes induced by Hebbian learning in the learning rule. However, weight changes induced by this learning rule can also cause weight changes in other synapses emanating from the same pre-synaptic neuron, even if they are not active. This would prove difficult to implement using the SpiNNaker framework described in section 2.3 as each synapse only has access to local information. Finally, both Potjans et al. (2011) and Frémaux et al. (2013) suggest that a more biologically plausible model of reward signals, modeled as a concentration of dopamine which gates and scales weight changes, also provides an effective model of TD learning.

### 4.2. Improving performance

As the results presented in section 3.3.1 show, due to the increased complexity of Algorithm 2 compared to Algorithm 1, the incoming spike processing performance of the three-factor STDP rule is approximately half that of the standard SpiNNaker STDP rule. While this is an unavoidable consequence of a more complex learning rule, if we wish to simulate our model in real-time, the only way to reduce the load on each core is to reduce the number of neurons being simulated on the core. This has the unfortunate side effect of also reducing the length of synaptic matrix rows which, as Figure 6 illustrates, reduces the efficiency of synaptic processing.

Knight and Furber (2016) developed an alternative method of mapping populations of neurons and their synapses to SpiNNaker which they called *synapse-centric mapping*. They split the time-driven simulation of neurons and the event-driven simulation of synapses between separate cores and these exchanged data using DMA transfers. This synapse-centric approach allows the processing of a synaptic matrix to be split between multiple cores in a row-wise manner. Unlike when the synaptic matrix is split in a column-wise manner—which occurs when the number of neurons per core is reduced using the approach discussed in this paper—this allows optimal synaptic matrix row lengths to be maintained. While Knight and Furber did not apply the synapse-centric approach to the three-factor STDP rule described in section 2.2, they demonstrated how it could be used to simulate highly-connected models using the spiking *Bayesian Confidence Neural Network* (BCPNN) learning rule (Tully et al., 2014) in real-time. BCPNN has similar properties to our three-factor STDP rule in that each synapse contains a trace as well as a synaptic weight and the cost of updating each synapse is significantly higher than for normal STDP. Therefore, we believe that combining the synapse-centric mapping with our three-factor STDP implementation would allow models with cortical levels of neuromodulated connectivity to be simulated in real-time—a significant improvement over the scaling properties illustrated in section 3.3.2.

### 4.3. Volume transmitters

Both chemical and electrical synapses are generally assumed to connect a pair of neurons in a one-to-one manner— Zoli et al. (1999) classifies this as *wired transmission*. However, there are also several *volume transmission* mechanisms used by the brain for one-to-many modes of communication. In areas of the brain with a high density of dopaminergic axons such as the striatum, dopamine is transmitted in a wired manner (Gerfen, 1988). However, Garris et al. (1994) showed that dopamine may also be transmitted extracellularly using volume transmission.

The method we have presented in this paper is well-suited to simulating wired dopamine transmission. However, if dopamine is delivered by volume-transmission, each synapses would receive spikes from all dopaminergic neurons within a volume with a radius of around 100 nm to 1 mm (Zoli et al., 1999). As Potjans et al. (2010) state, this means that each synapse would be likely to receive substantially more dopaminergic than pre-synaptic spikes. Potjans et al. propose a novel approach for simulating such synapses on a distributed system where separate nodes handle the dopaminergic spikes arriving at each machine running the simulation. These nodes are responsible for sorting the dopaminergic spikes and delivering them, when requested by the equivalent of Algorithm 2, to the nodes simulating the synapses. Additionally, the volume transmitter nodes send dopaminergic spikes to the nodes simulating the synapses at regular intervals, minimizing the amount of memory required for dopaminergic spike storage. Potjans et al. demonstrated this approach by building a model consisting of 1 × 10^5^ neurons and 1 × 10^9^ synapses – each of which received a total neuromodulatory spike rate of 500 Hz. They showed that, using their new approach, simulations of this model exhibited supralinear scaling up to 32 machines and, beyond that, linear scaling up to 1,024 machines.

In the context of SpiNNaker, the large numbers of dopaminergic spikes in the post-synaptic history structure that would result from simulating volume transmitters using the approach we presented in section 2.3 would be even more problematic. Firstly, Figure 6 suggests that the spike handling performance of our implementation would be very low if each synapse received neuromodulatory spikes at the rates used in the model developed by Potjans et al. Secondly, the NEST simulator used by Potjans et al. stores post-synaptic history in a dynamic data structure (described in detail by Morrison et al., 2007), whereas, due to each core's limited local memory, SpiNNaker uses a static data structure. Therefore, if the number of post-synaptic or dopaminergic spikes increases beyond the fixed capacity of this structure, spikes will not be processed and simulation results will be incorrect. We believe that the approach developed by Potjans et al. could be adapted to solve these issues by using one core on each SpiNNaker chip to manage the gathering of neuromodulatory spikes and delivering them by DMA to the cores responsible for simulating the neuromodulated STDP synapses. This core could also be responsible for performing the regular, time-driven weight updates due to dopaminergic spikes, perhaps using a similar approach to that proposed by Galluppi et al. (2015).

### 4.4. Robotics

One interesting future direction for this work would be to implement a reinforcement learning agent which could perform instrumental conditioning tasks using the SpiNNaker implementation of dopamine modulated STDP presented in this paper. Shim and Li (2017) did some work in this area and presented a collision avoidance agent using the same learning rule that we have implemented. However, they only tested these agents in a simulated environment whereas, using SpiNNaker, it would be possible to simulate the spiking neural network based controller in real-time so it could be evaluated, embodied in a real robot.

## Author contributions

JK: Developed the mathematical model; MM and JK: Developed and benchmarked the learning rule; GP: Developed the Pavlovian conditioning experiment; MM, JK, GP, and SF: Wrote the paper; SF: Provided supervision.

### Conflict of interest statement

The authors declare that the research was conducted in the absence of any commercial or financial relationships that could be construed as a potential conflict of interest.
